The article "The use of surrounding rock loosening circle theory combined with elastic-plastic mechanics calculation method and depth learning in roadway support" was retracted in 2024. Reasons: duplicate publication; overlap with earlier publications; compromised peer review; unreliable results or conclusions.

# The use of surrounding rock loosening circle theory combined with elastic-plastic mechanics calculation method and depth learning in roadway support

**DOI:** 10.1371/journal.pone.0234071

**Published:** 2020-07-15

**Authors:** Qingyun Xu, Yongming Li, Jie Lu, Lei Zhang

**Affiliations:** School of coal engineering, Shanxi Datong University, Datong, Shanxi, China; University College London, UNITED KINGDOM

## Abstract

The objective is to study the design method of roadway support and provide technical support for coal mining and other mining methods that need deep roadway excavation. Through literature review, the occurrence, development mechanism and influencing factors of surrounding loose rock zones of roadways are analyzed. A method of detecting is selected according to the characteristics of surrounding rock loosening. Knowledge of elastoplastic mechanics is used to theoretically study the failure mechanism of surrounding rock in deep re-mining roadways. Based on the artificial neural network prediction model (ANN), the surrounding rock is classified and a support network model of the decision system is constructed. After the design of roadway support, a sharp change of vault subsidence normally occurs within about 7 days after excavation, and the total subsidence is 14 mm. In the following month, deformation is slow, subsidence is small, and it is basically stable after one month. The curve of the vault subsidence rate shows that the vault subsidence rate is less than or equal to 1mm/d after 7 days. The convergence rate is also less than 1 mm/d after 7 days. There are two cave mouths AB and CD, and the convergence value of AB is 6.47mm, CD is 10.26mm: CD is slightly larger than AB, and it is close to stable one month later. It is essentially consistent with the time of vault settlement and stability, and the amount of deformation is approximately the same. This shows that, with the advance of the working face, the displacement of the surrounding rock in the section away from the working face will gradually decrease and the surrounding rock will be stable. The stability time of surrounding rock displacement of the portal section is the same as that of vault subsidence under the initial support, and the amount of deformation is approximately the same, indicating that the support parameters and construction methods are reasonable.

## 1. Introduction

China is the country with the highest coal output in the world and is heavily dependent on coal resources. However, due to China’s rapid development, the demand for coal resources is still increasing. Until the best alternative energy source is found, coal will always be used as the main source of energy in China. However, because of increased coal mining, there are few remaining coal resources that are easy to mine, so coal mining in China needs to extend deeper underground [1].

As coal mining becomes deeper, the difficulty of mining increases rapidly and greater demands are made of coal mining technology and roadway support technology. The greater the mining depth is, the more difficult the roadway support is, and the lower the stability of the roadway is. Hence, research on the new roadway support method is urgent [2]. With the emergence of a new roadway support mode, new support theory has emerged, while the current support theory has reached its limits.

In recent years, most coal mining has entered the deep mining stage. In the new geological situation, the existing single roadway support method cannot meet the current requirements for maintaining the stability of the roadway [3]. Therefore, in view of the problems existing in roadway support, the method of combined support has been studied. The method of combined support is not simply to stack the existing single roadway support method many times, but to coordinate the various support components and characteristics of the existing method, so as to develop the support capability beyond that of the single roadway support method. For example, at present, the popular combined support method of anchor, mesh and cable integrates the three support means of bolt support, anchor cable support and anchor mesh support to prevent the deformation of the surrounding rock to the maximum extent and maintain the stability of the roadway [4].

Already, scholars at home and abroad have carried out extensive theoretical research and practical tests on underground excavation engineering, and developed a variety of support theories. Moreover, most of these tests have been undertaken in productive coal mines and achieved good results. At the same time, the rapid development of various mechanics disciplines is very helpful for the study of rock mass properties, rock failure mechanisms and roadway support theory in underground engineering [5].

Some scholars believe that roadway support should be focused on the main bearing area, because the main bearing area plays a major role in the control of surrounding rock deformation, while the secondary bearing area plays an auxiliary role [6]. After the excavation of the roadway, the stress of the surrounding rock is redistributed, a compression zone is formed in the depths of the surrounding rock, and a tension zone is formed near the roadway. The former is called the main bearing area, and the latter is the secondary bearing area.

Some scholars put forward the theory of “surrounding rock loosening circle” according to the relationships in the size of the surrounding rock loosening circle. In this theory, it is considered that, when the roadway is excavated in hard surrounding rock, the surrounding rock of the roadway will not deform obviously when there is no supporting structure, because the size of the surrounding circle of loosening rock is close to zero at this time [7]. However, when the surrounding rock is not hard, the loose zone of surrounding rock will gradually increase with time. The convergence deformation of the larger loosening circle will increase, which is reflected in the increase of deformation of the surrounding rock, increasing the difficulty of supporting the roadway. Therefore, the essence of roadway support is to limit the unfavorable deformation of the surrounding rock loosening circle as it increases [8].

In this study, through literature review, the occurrence, development mechanism and influencing factors of the surrounding rock loosening circle of roadways are analyzed. A detection method is selected according to the characteristics of the surrounding rock loosening. Knowledge of elastoplastic mechanics is used to study the failure mechanism of surrounding rock in deep re-mining roadways. Based on the artificial neural network prediction model (ANN), the surrounding rock is classified and a support network model of the decision system is constructed. Numerical simulation and field observations of roadway deformation are used to verify the decision system.

## 2. Method

### 2.1 Mechanical model of roadway surrounding rock

There are many forms of failure of surrounding rock around a roadway. In different locations and different failure stages, the forms of failure are also different. According to the specific form, process and cause of the surrounding rock failure of the roadway, it can be roughly divided into the following types: local rockfall failure, tension failure and bending failure, heavy shear failure, shear failure and composite failure, rock burst failure, deliquescence expansion failure [9].

The stability of rock surrounding a roadway is relative. The concept of stability differs, depending on the production field and use requirements. Generally speaking, surrounding rock instability refers to the phenomenon of surrounding rock failure or extensive deformation that hinders production or safety, such as roof collapse, two sides of extrusion, floor uplift, surrounding rock cracking, rock burst, shotcrete crack or support damage: none of these should occur. However, the concept of stability of the rock surrounding a roadway is different, depending on specific standards or requirements [10].

For example, mudstone, shale, claystone, tuff, marl, and other rocks are easy to form swelling and deliquescence. This kind of expansive rock stratum will expand rapidly after absorbing water since it contains a lot of active minerals. In addition, the existence of rheological property will cause the strength of the swelling rock decreased or even disappeared, because this kind of rock is more easily affected by weathering, deliquescence, softening, and argillization. Thus, the surrounding rock roadway should be supported in time after excavation, and measures such as spraying layer should be taken to isolate the surrounding rock from water and air, thereby preventing its deliquescence and expansion damage.

Under the condition of deep mining, both the original rock stress and the self-weight stress of rock mass are very large. When the roadway is excavated, with the original balanced state of stress being broken, the surrounding rock will inevitably be damaged. A new relationship of mechanical equilibrium will eventually form again around the surrounding rock. At this time, there will be several areas with significantly different mechanical relations. From the degree of damage of surrounding rock, it can be divided into three areas; namely, crushing area, plastic area and elastic area, as shown in Fig 1.

**Fig 1:** Distribution of stress state of rock.

Divide the cave mouths into AB and CD sides as shown in Fig 1.

According to the stress state of the surrounding rock, ways of supporting the surrounding rock can be determined: bolt support or anchor cable support. The function of an anchor bolt is basically the same as that of an anchor cable support. The unstable rock layer can be fixed to a stable rock layer through external action, thus achieving support. Different support methods should be selected for different degrees of stability of the surrounding rock.

The bottom extraction roadway of a coal mine is selected as an example to carry out the industrial test of "the stability classification and support decision system of the surrounding rock of the deep roadway".

The strata in this area are nearly monoclinic structure, which from the bottom to the top are light-gray fine sandstone, gray coarse siltstone, silver-gray recruit mudstone, and gray-white fine sandstone, showing gentle wave bedding, gray fine siltstone, gray-white fine sandstone, and gray mudstone. The hydrogeological conditions in this area are relatively simple. The main underground water source is sandstone fissure water at the top and bottom plates, and it is predicted that there is water pouring and seepage at the local lithologic fracture.

### 2.2 Detection of the loose zone of surrounding rock

For research on the loosening and stability of the rock surrounding roadways, the existing research results mostly divide the rock surrounding a roadway into an elastic area, a plastic area and the most internal fracture area. There are some mature theories about the solution of the elastic zone and the plastic zone. However, for the size of the broken zone, there is still no conclusion on the theoretical calculation to be carried out. Although there are some formulas for calculating the fracture area, there is a big gap between the quantitative analysis and the actual situation, due to insufficient understanding of the properties of rock after fracture in the fracture area.

The main reason for this is that there is a big gap between some basic assumptions of the existing calculation theory and the actual state of the surrounding rock [11]. The roadway loose zone is a broken zone formed around the roadway when the stress of the surrounding rock exceeds the strength of the rock mass. Its physical state shows an increase in fracturing and a decrease in the rock stress level. The loose circle test is to detect the new cracks and their distribution range after excavation. The interface with and without fracture in surrounding rock is the boundary of the loosening circle [12]. In the field, the thickness of the loose area can be measured by the acoustic wave method, the multi-point displacement meter method or the GPR method.

The ultrasonic testing technology of the roadway surrounding rock-loosening circle uses the correlation between the propagation parameters (time value, velocity, amplitude, attenuation coefficient, etc.) of ultrasonic waves in the geotechnical medium and structure and the physical and mechanical indexes (dynamic modulus, density, strength, etc.) of the geotechnical medium and structure.

Based on the elastic theory, the relationship between the velocity of ultrasonic longitudinal waves and the elastic parameters of the medium can be obtained from the wave equation of elastic waves through the derivation of the static equation of the spatial problem of elastic mechanics [13].

$$V_{p}=\sqrt{\frac{E}{\rho }\cdot \frac{1-v}{\left(1+v)(1-2v\right)}}$$ (1)

$$V_{s}=\sqrt{\frac{E}{\rho }\cdot \frac{1}{2(1+v)}}$$ (2)

In the equation, *ρ* is density, E is modulus of elasticity, and v is Poisson's ratio.

Because of the different rock, rock mass and structure, its physical parameters are different, so its propagation speed is also different. Conversely, the situation of rock and rock mass can be distinguished according to the sound wave propagation speed of the rock mass.

### 2.3 Mechanical calculation of elastoplasticity

1) The change of stress and displacement in the elastic zone;

(1) Basic mechanical equation of the elastic zone;

According to the theory of elastoplasticity, there are several basic equations for the asymmetry in plane strain problems:

Equilibrium differential equation:

$$\frac{d\sigma_{r}}{dr}+\frac{\left(\sigma_{r}-\sigma_{0}\right)}{r}=0$$ (3)

Geometric equation:

$$\begin{array}{l} \varepsilon_{r}=\frac{du}{dr}\\ \varepsilon_{0}=\frac{u}{r} \end{array}\}$$ (4)

Deformation compatibility equation:

$$\begin{array}{l} \frac{d\varepsilon_{0}}{dr}+\frac{1}{r}(\varepsilon_{0}-\varepsilon_{r})\\ \varepsilon_{r}=\frac{1-\mu^{2}}{E}(\sigma_{r}-\frac{\mu }{1-\mu }\sigma_{\theta })\\ \varepsilon_{\theta }=\frac{1-\mu^{2}}{E}(\sigma_{\theta }-\frac{\mu }{1-\mu }\sigma_{r}) \end{array}\}$$ (5)

In these equations, u is the radial displacement of the surrounding rock of the roadway, which is positive towards the roadway, otherwise negative; *σ*_*r*_ and *σ*_0_ are the radial and tangential stresses of the rock surrounding the roadway; *ε*_*r*_ and *ε*_*θ*_ are the radial and tangential strains of the surrounding rock of the roadway; r is the distance from the circular roadway; E is the modulus of elasticity; *μ* is Poisson's ratio.

(2) Boundary conditions;

When the outer boundary of the elastic region approaches infinity, it has the following relations:

$$\sigma_{r}=\sigma_{\theta }=P_{0}$$ (6)

The inner boundary of the elastic region is set as r = R_P_. At the boundary of the elastic and plastic zones, the condition of elastic asymmetry should be satisfied. According to the Coulomb strength limit criterion:

$$\sigma_{0}=K\sigma_{r}+\sigma_{c},\;and\;\sigma_{r}+\sigma_{0}=2P_{0}.$$

Where, K is the stress coefficient, and $K=\frac{1+\sin\theta }{1-\sin\theta }$.

P_0_ is the original rock stress.

*σ*_*c*_ is the uniaxial compressive strength of the rock, and $\sigma_{c}=\frac{2c\cos\theta }{1-\sin\theta }$.

C is rock cohesion.

At the same time, there are continuity equations of stress and displacement at the inner boundary of elastic region.

$$\begin{array}{l} \sigma_{r}^{P}=\sigma_{r}^{c}=\sigma_{r}^{R_{p}}=\frac{2KP_{0}-\sigma_{c}}{K+1}\\ \sigma_{\theta }^{P}=\sigma_{\theta }^{c}=\sigma_{\theta }^{R_{p}}=\frac{2KP_{0}+\sigma_{c}}{K+1} \end{array}\}$$ (7)

, $\sigma_{r}^{P}$ and $\sigma_{0}^{P}$ are the radial stress and tangential stress at the boundary of the elastic zone;

$\sigma_{r}^{c}$ and $\sigma_{0}^{c}$ are the radial stress and tangential stress at the boundary of the plastic zone;

$\sigma_{r}^{R_{p}}$ and $\sigma_{\theta }^{R_{p}}$ are the radial stress and tangential stress at the boundary of elastic-plastic zone.

2) Stress change and displacement equation in plastic zone;

(1) Basic equation;

The equilibrium differential equation and the geometric equation are the same as those in the elastic region. In the plastic zone, according to the Coulomb criterion, the stress limit state equation can be obtained as follows:

$$\sigma_{\theta }=K\sigma_{r}+\sigma_{c}^{P}$$ (8)

Where the uniaxial compressive strength $\sigma_{c}^{P}$ of surrounding rock in the plastic zone meets $\sigma_{c}\geq \sigma_{c}^{P}\geq \sigma_{c}^{*}$. Moreover, it has the following relationship with strain:

$$\sigma_{c}^{P}=\sigma_{c}-M(\varepsilon_{\theta }-\varepsilon_{\theta }^{c})$$ (9)

Where, M is the plastic correlation coefficient, M = tan θ.

$\varepsilon_{\theta }^{c}$ is the strain of surrounding rock at peak value.

(2) Boundary conditions;

The boundary here mainly refers to the inner and outer boundaries of the plastic zone. Inner boundary refers to the boundary between the plastic zone and the broken zone, which is recorded as R_b_. It is not only the inner boundary radius of the plastic zone, but also the outer boundary radius of the broken zone. The outer boundary refers to the inner boundary of the elastic region.

3) The change of stress and displacement in the broken zone;

(1) Basic equations of mechanics;

The basic elastic-plastic equations in the broken zone are the same as those in Eqs (1) and (2).

The limit-state equation in the broken zone can be obtained according to the Coulomb criterion:

$$\sigma_{\theta }=K\sigma_{r}+\sigma_{c}^{*}$$ (10)

Where, $\sigma_{c}^{*}=\frac{2C^{*}\cos\theta^{*}}{1-sin\theta^{*}}$.

$\sigma_{c}^{*}$ represents the uniaxial compressive residual strength of the surrounding rock in the broken area;

C* represents the residual cohesion of the surrounding rock in the broken area;

and θ* represents the internal friction angle of the surrounding rock in the broken area.

(2) Boundary conditions in the broken zone;

When r = R_b_, it is the outer boundary of the broken zone, which is also the inner boundary condition of the plastic zone of the surrounding rock.

When r = R_0_, it is the inner boundary of the broken zone.

In these equations, *σ*_*r*_ = p_1_, where p_1_ is the surrounding rock support force.

4) Discussion of the solution;

(1) Based on the above analysis of elastic-plastic mechanics, it can be concluded that, in the situation of deep re-mining, the deformation of the surrounding rock of the roadway mainly comprises of deformation in the elastic zone (U^c^), deformation in the plastic zone (U^p^) and deformation in the broken zone (U^b^). Through mathematical processing, the relationship between the change of the crushing area and the deformation of the roadway can be obtained as follows:

$$u=\frac{2p^{'}r_{0}}{E}\left\{C_{1}\left[\frac{n_{2}}{m_{1}n_{1}}+\frac{1}{n_{1}}{\left(1+\frac{L_{b}}{r_{0}}\right)}^{n_{1}}\right]\right\}$$ (11)

From the relationship, it is not difficult to find that the deformation u of the roadway changes in a positive proportion to L_b_, but has little relationship with r_0_; that is to say, the deformation of the roadway is mainly affected by the thickness of the broken area and has little relationship with the size of the plastic area. The larger the broken area, the larger the deformation of the deep re-mining roadway.

(2) Under certain mining conditions (mainly referring to a certain mining depth and roadway section), the size of the surrounding rock fracture area of the deep re-mining roadway is mainly affected by support resistance and residual strength.

(3) In order to reduce the deformation of the deep re-mining roadway, it is necessary to increase the support resistance of the roadway support and increase the residual strength of the surrounding rock in the broken area.

### 2.4 Realization of roadway support based on deep learning

Deep learning is a new field in machine learning research. Its motivation is to build and simulate the neural network of the human brain for analysis and learning. It mimics the mechanism of the human brain to interpret data, such as images, sounds, and text. Deep learning is a kind of unsupervised learning. The concept of deep learning comes from research into ANN. Multilayer perception with multiple hidden layers is a kind of deep learning structure. Deep learning, by combining low-level features to form more abstract high-level representation of attribute categories or features, is used to discover the distributed feature representation of data.

ANN is an artificial network composed of many processing units which are widely interconnected. It is used to simulate the structure and function of the brain and nervous system. These processing units are called artificial neurons. ANN can be regarded as a directed graph, with artificial neurons as nodes and connected by directed weighted arcs.

Neural networks simulate the brain in two ways:

First, the knowledge acquired by a neural network is learned from the external environment.

Second, the connection strength of internal neurons, i.e., synaptic weight, is used to store the knowledge acquired.

The main task of a neural network is to establish the model and determine the weight. Generally, there are two kinds of network structures; the forward type and the feedback type. The learning and training of a neural network needs a group of input data and output data pairs. After selecting the network model and transfer and training functions, the neural network calculates the output results, and corrects the weight according to the error between the actual output and the expected output. When the network judges, only the input data but not the expected output results are needed. A very important ability of neural networks is that a network can learn from the environment through the constant adjustment of its neuron weight and threshold value, until the output error of the network reaches the expected result, and then it is considered that the network training is over.

The full name of the BP algorithm is the “error back propagation algorithm”. The basic idea of the algorithm is: in the feedforward network, the input signal is input through the input layer and output through the hidden layer calculation. The output value is compared with the marked value. If there is any error, the error is propagated from the output layer to the input layer in the reverse direction. In this process, the neuron weight is adjusted by the gradient descent algorithm. The BP neural network (BPNN) is such a neural network model, which is composed of one input layer, one output layer, and one or more hidden layers. Its activation function is a sigmoid function, and its multilayer feedforward neural network is trained by the BP algorithm.

The specific steps of the BP algorithm are as follows. Where O represents the neuron, net represents the network, E represents the mean square error between the actual output and the expected output, and w represents the network weight.

1) Forward: find the output of all neurons.

$$net_{j}=\sum_{i}w_{ij}O_{i}$$ (12)

$$O_{j}(k)=f(net_{j})$$ (13)

2) The mean square error between the actual output and the expected output is calculated.

$$E=\frac{1}{2}\sum_{j}{\left(y_{j}-{\hat{y}}_{j}\right)}^{2}$$ (14)

3) Reverse: for each node, calculate the partial derivative (gradient) of error to weight.

$$\frac{\partial E}{\partial w_{ij}}=\frac{\partial E}{\partial net_{j}}\cdot \frac{\partial net_{j}}{\partial w_{ij}}=\delta_{j}(k)\cdot O_{i}$$ (15)

4) Use iterative equation to update network weight.

$$w_{ij}(k+1)=w_{ij}(k)=\delta_{j}(k)\cdot O_{i}(k)$$ (16)

5) Judge whether to continue or end the iteration.

### 2.5 Overall structure of the system

The design of a roadway support decision-making system can be divided into the following modules:

(1) BPNN: use BPNN to analyze many factors affecting roadway support, and get specific roadway support results;

(2) surrounding rock classification: Based on the detection of the loosening ring of surrounding rock, use the surrounding rock classification module to classify the surrounding rock;

(3) roadway support design: according to the data obtained from the first two modules, carry out the specific support design.

The various modules of the decision support system are not isolated, but have internal relations with each other. The flow chart of the modular design of the system is divided in detail, as shown in Figs 2 and 3.

**Fig 2:** Neural network model training flow chart.

**Fig 3:** Flow chart of stability classification module of surrounding rock.

Figs 2 and 3 show that each module is both independent and linked. All modules together constitute the decision system of roadway support design, but each module works separately, greatly improving the working efficiency of the decision system of roadway support.

Input the data of the roadway to be supported into the BPNN module, and get the corresponding bolt parameters, anchor cable parameters, spray layer, and mesh parameters through the training of the BPNN module, and classify the roadway to achieve its stability, thus designing the support of the roadway.

## 3. Results and discussion

### 3.1 Design results of support decision system

According to the relevant information and quantitative index of the surrounding rock in the bottom extraction roadway, the "stability classification and support decision system of the surrounding rock in the deep shaft" was used to enter the surrounding rock stability classification interface. Each group of data was input to the corresponding position of the software window. The trained neural network was opened and the simulation was started to classify the surrounding rock of the roadway. After the simulation, the results were saved. After returning to the system menu option, the roadway support optimization design interface was accessed and the system automatically imported the related data to simulate the process of roadway surrounding rock stability classification. The dimension data of the straight-wall, semi-circular arch roadway was input and the support design system generated the basic support parameters.

After the support design was completed, the basic design parameters of the roadway were displayed in the form of text documents. In the design result interface of rolling support, the corresponding design section of roadway support was displayed.

### 3.2 Data monitoring of portal section

In order to verify the effect of applying the support decision system, the surrounding rock displacement and vault subsidence of the portal section were analyzed. The change curve and rate of vault settlement are shown in Fig 4.

**Fig 4:** Curve of vault subsidence and change of subsidence rate.

The curve of crown subsidence shows that the sharp change of crown subsidence mainly occurs within about 7 days after excavation, and the total subsidence is 14 mm. In the following month, the deformation is slow and the subsidence is small. After one month, it is close to stable. The curve of the vault subsidence rate shows that the vault subsidence rate is less than or equal to 1mm/d after 7 days.

The convergence value and convergence rate of the AB edge of the portal are shown in Fig 5. The convergence value and convergence rate of the CD edge of the portal are shown in Fig 6:

**Fig 5:** Curve of convergence and convergence rate of AB side of portal.

**Fig 6:** Curve of convergence and convergence rate of CD side of portal.

Figs 5 and 6 show that the sharp convergence around the portal is about 7 days, and the convergence rate is less than 1mm/d after about 7 days. The convergence value of AB is 6.47mm, CD is 10.26mm: CD is slightly larger than AB, and it is close to stable one month later. The settlement time is essentially the same as that of the vault, and the deformation is approximately the same. This shows that, with the advance of the working face, the displacement of the surrounding rock in the section away from the working face will gradually decrease and the surrounding rock will be stable.

The stability time of the surrounding rock displacement of the portal section is almost the same as that of vault subsidence under the initial support, and the amount of deformation is approximately the same, which shows that the support parameters and construction methods are reasonable;

The influencing factors of deformation and instability of roadway and support are obtained, and the selection principle of corresponding support design index is also given. Based on the theory of surrounding rock loosening circle and elastic-plastic theory, this study provides the basis for the decision-making system. Based on the depth learning prediction model, the decision-making system and support network model are constructed.

## 4. Conclusion

In situations of deep mining, the stability of re-mining roadways differs greatly from the shallower part. The roadway is easy to break, difficult to maintain and has large deformation. At the same time, under the deep mining conditions, the structural stress and self-weight stress of the surrounding rock of the roadway are significantly increased, which increases the difficulty of support. The traditional roadway support method cannot be adapted to the deep re-mining roadway, but the new "bolt mesh cable" combined support method lacks relevant theoretical research in the deep re-mining environment.

Through a literature review, the occurrence, development mechanism and influencing factors of the surrounding rock loosening circle of the roadway are analyzed. A detection method is selected according to the characteristics of surrounding rock loosening. Knowledge of elastoplastic mechanics is used to study the failure mechanism of surrounding rock in a deep re-mining roadway. Based on the artificial neural network prediction model, the surrounding rock is classified and a network model of the support decision system is constructed.

Numerical simulation and field observations of roadway deformation are used to verify the decision system. The test results show that the support decision-making system in this study has strong practicability and reliability, which can provide a basis for roadway support construction. Due to the limitation of time and theoretical level, there are still many deficiencies in the support decision-making system, which will be further improved in future research. Other excellent programming languages, such as C, could be combined to optimize the system in depth. Due to time, there are no other supporting methods in the sample, such as shed, section grouting, etc. If these are used, it will be necessary to add samples and redesign the system interface.

## Supporting information

S1 Data (XLS)
